# On the effect of vitamin C intake on human health: How to (mis)interprete the clinical evidence

**DOI:** 10.1016/j.redox.2020.101532

**Published:** 2020-05-23

**Authors:** Jens Lykkesfeldt

**Affiliations:** Faculty of Health & Medical Sciences, University of Copenhagen, DK-1870, Frederiksberg C, Denmark

## Abstract

For decades, the potential beneficial effect of vitamin C on human health—beyond that of preventing scurvy—has been subject of much controversy. Hundreds of articles have appeared either in support of increased vitamin C intake through diet or supplements or rejecting the hypothesis that increased intake of vitamin C or supplementation may influence morbidity and mortality. The chemistry and pharmacology of vitamin C is complex and has unfortunately rarely been taken into account when designing clinical studies testing its effect on human health. However, ignoring its chemical lability, dose-dependent absorption and elimination kinetics, distribution via active transport, or complex dose-concentration-response relationships inevitably leads to poor study designs, inadequate inclusion and exclusion criteria and misinterpretation of results. The present review outlines the differences in vitamin C pharmacokinetics compared to normal low molecular weight drugs, focusses on potential pitfalls in study design and data interpretation, and re-examines major clinical studies of vitamin C in light of these.

## 1 Introduction

Countless clinical studies have investigated the effects of vitamin C on human health ever since the identification of its role in the prevention of scurvy. These can roughly be divided into i) mechanistic studies investigating the pharmacokinetics of vitamin C, its homeostasis and the role of ascorbate in various physiological processes, ii) epidemiological studies exploring associations between vitamin C intake or status and morbidity and mortality, and finally iii) intervention studies examining the effect of vitamin C supplementation on disease prevention, progression and treatment. Despite this wealth of scientific evidence, some very basic albeit fundamental questions remain unanswered to this day including: “*What is the optimal intake of vitamin C?”* and “*What is the preventive and therapeutic potential of vitamin C?”*

A major reason for the continued controversies about the putative importance vitamin C in human health can be found in the interpretation and quality of the available clinical data. Randomized controlled trials (RCTs) are generally considered the gold standard in drug efficacy and safety testing. Naturally, the RCT paradigm has been applied to micronutrient studies in search of clinical support for a possible functional health benefit of dietary supplementation. For vitamin C, such intervention studies have with few exceptions been unsuccessful showing only minor or no effects on morbidity and mortality [1]. However, vitamin C differs significantly from the typical low molecular weight pharmaceutical drug in a number of ways that need to be incorporated into study designs and interpretation to achieve valid conclusions [2]. Epidemiological studies on the other hand are often accused of suffering from potential selection bias and confounding. Moreover, their lack of ability to establish causality and discriminate between multiple etiological sources may suggest the possibility that identified associations be merely coincidental or secondary with respect to vitamin C status *per se* [3].

As humans do not have the capacity to synthesize vitamin C in contrast to the vast majority of mammalian species, its pharmacokinetics has been devoted particular attention as a basis for the evaluation of uptake, distribution, metabolism and clearance. Other species potentially have the capacity to increase biosynthesis of vitamin C in times of need. However, in humans, increased turnover—due to e.g. diseased-induced inflammation or oxidative stress—can only be compensated by increased intake or by supplementation.

One important aspect of dose selection in intervention studies is the assumption of near 1st order kinetics within the therapeutic range. For vitamin C, convincing data were published decades ago indicating that vitamin C pharmacokinetics is in fact highly dose-dependent in humans within the physiological range [4,5]. Despite this important breakthrough, the consequences of these observations and the true complexity of vitamin C homeostasis did not become evident until the identification of the sodium-dependent vitamin C transporters (SVCTs). The SVCTs are now considered the primary means of systemic control of vitamin C homeostasis and are capable of actively transporting ascorbate into cells against a considerable concentration gradient [6]. The resulting dose-dependency and non-linearity of the pharmacokinetics profoundly changes fundamentals of study design and data interpretation but unfortunately, this reality has mostly been neglected in the clinical vitamin C literature.

While not attempting to answer the highly pertinent questions listed above as insufficient evidence is available, the purpose of this review is to discuss the pharmacology of vitamin C and to critically re-examine the larger studies from the clinical literature on vitamin C in light of the potential pitfalls that may lead to misinterpretations.

## 2 Pharmacokinetics of vitamin C

The pharmacokinetics of vitamin C has recently been reviewed in detail [7] and only a brief overview is provided here. The intestinal absorption of orally ingested vitamin C—that being from food sources or supplements alike—occurs through transporter proteins rather than by passive diffusion [8,9]. Several decades ago, it was observed by independent investigators that increasing oral doses beyond 200–400 mg vitamin C/day leads to decreasing absorption fractions and it was concluded that intestinal vitamin C absorption is subject to saturable active transport [4,5]. Levine and coworkers later performed a series of meticulous pharmacokinetic studies in healthy young men and women showing that plasma saturation occurs at a concentration around 70–80 μM [10,11] (Fig. 2H). Other studies have arrived at the same number [12,13]. This phenomenon also accounts for the highly different pharmacokinetics of vitamin C following oral vs. parenteral administration (reviewed in more detail in Ref. [7]). It became known that dehydroascorbic acid (the oxidized form of vitamin C) has the ability to pass through a number of glucose transporters by facilitated diffusion [[14], [15], [16], [17]], but this realization did not explain the dose-dependency following oral ingestion. Later, it was discovered that ascorbate (the reduced form of vitamin C) and dehydroascorbic acid are taken up by separate mechanisms in the intestine and that uptake of ascorbate is sodium dependent [18]. This coincided with the discovery and characterization of the sodium-dependent vitamin C transporter (SVCT) family by Tsukaguchi and coworkers [6], who later found that the intestine contains the low affinity/high capacity active transporter SVCT1 [19]. Moreover, SVCT1 is also present in the epithelium of the proximal renal tubuli and governs the active reabsorption of ascorbate in the kidneys [19]. It has been shown in *Slc23a1*^*−/−*^ mice lacking the SVCT1 that renal fractional excretion increases up to 18-fold, while intestinal absorption is not significantly diminished [20]. This suggests that the renal SVCT1-mediated reabsorption of ascorbate is pivotal in the maintenance of systemic vitamin C homeostasis. The active transporter displays dose-dependency and its expression may be regulated by vitamin C status in several tissues [8,21,22].

Several single-nucleotide polymorphisms (SNPs) have been identified in the human SVCT1. Most of these are suggested to lead to a lower homeostatic set point, but reliable data on vitamin C kinetics from these subpopulations are difficult to obtain due to the rare occurrence of some of the individual SNPs and so far, very limited data are available. However, a few studies have suggested that such SNPs may be linked to increased disease risk. Thus, Zanon-Moreno et al. found significant associations between the rs1279386 SNP in SLC23A2 and lower plasma vitamin C concentrations as well as increased risk of glaucoma [23]. SNP rs6596473 of SLC23A1 has been suggested to be associated with aggressive periodontitis [24]. Kobylecki et al. investigated a SNP rs33972313 that provide higher vitamin C concentration than the wildtype in a Mendelian randomization study of cardiovascular mortality and morbidity. They concluded that their data “cannot exclude that a favorable effect of high intake of fruit and vegetables could in part be driven by high vitamin C concentrations” [25]. In other words, although the data were not conclusive, they indicated that the SNP could be associated with improved cardiovascular health. Interestingly, Corpe et al. modelled dose vs. concentration curves for a selected number of known SNPs and found that the functionally poorest SVCT allele identified (A772G, rs35817838) was expected to result in a plasma saturation level corresponding to life-long vitamin C deficiency [20]. However, these modelling studies and their potential phenotypic consequences remain to be confirmed in clinical studies.

Distribution of vitamin C from plasma to tissues are primarily governed by the SVCT2, i.e. the low-capacity high-affinity version of the vitamin C transporter. It is located in most cell types and it appears that local concentrations and/or isoforms of the transporter determine the steady state concentration of the individual organ/tissue [7]. From detailed studies in guinea pigs (that like humans are unable to synthesize vitamin C), it is known that differences in expression levels of SVCTs leads to a highly diverse distribution of vitamin C between organs (See Fig. 1) [21,22]. Thus, up to 20-fold difference in steady state concentration has been measured between e.g. brain/adrenal gland and kidney/heart/muscle being among tissues with the highest and lowest in steady state concentrations, respectively [[26], [27], [28], [29], [30], [31]].

**Fig. 1:** Distribution of vitamin C is highly differential between organs of the body. Several organs have concentration-dependent mechanisms for retention of vitamin C maintaining high levels during times of inadequate supply at the expense of other organs. Particularly protected is the brain. In addition, the concentration-dependent absorption and re-absorption mechanisms contribute to the homeostatic control of the vitamin C in the body. Reproduced from Ref. [7].

**Fig. 2:** Comparison of vitamin C and an average low molecular weight drug with regard to plasma concentration. Left panels illustrates intravenous administration, right panels oral administration, respectively. Schematic plasma concentration vs time following a bolus and maximal plasma concentration vs dose plots are compiled from data in Refs. [7,10,11,27,48,49,54,[94], [95], [96], [97]]. Plots are approximations for illustrative purposes only. **A:** An average drug displays 1st order kinetics following i. v. administration with a constant elimination half-life. **B:** Oral administration gives rise to an absorption phase followed by a 1st order elimination with a half-life similar to that of i. v. administration. **C:** Intravenous administration of vitamin C typically results in 1st kinetics until the physiological concentration range is reached where the elimination will gradually decline. **D:** The effect of oral administration of vitamin C on the plasma concentration will depend considerably on the vitamin C status of the individual. Vitamin C deficiency will promote quantitative uptake while vitamin C sufficiency will promote excretion with little impact on the plasma concentration profile. **E & F:** For the average drug, the maximal plasma concentration is proportional to the dose regardless of route of administration. **G:** A recent compilation of i. v. data revealed that the maximal plasma concentration following i. v. administration of vitamin C is proportional to the (infusion) dose up to about 50 mmol/L (corresponding to a dose of 70 g/m^2^ after which is does not increase further [7]. H: Plasma C_max_ following oral administration of vitamin C is not proportional to the dose but displays saturation kinetics [11,98].

Metabolism of vitamin C is intimately linked to its redox status. Ascorbate is an efficient chain-breaking antioxidant both capable of quenching free radicals and specifically donating electrons to a considerable number of mono- and dioxygenase enzymes [32]. Moreover, a whole range of mechanisms has evolved to ensure that oxidized vitamin C is almost quantitatively salvaged by intracellular recycling of its oxidized form back to the biologically active reduced form ascorbate by a variety of cell types [[33], [34], [35], [36], [37], [38], [39], [40], [41], [42]]. Thus, the daily turnover of vitamin C in healthy non-smoking individuals has been estimated to a mere 3% [43], thereby grossly limiting the daily amount necessary to be ingested to maintain sufficiency. Moreover, it has been estimated in both in vitro and in vivo studies that erythrocytes are capable of recycling the total amount of vitamin C present in blood approximately once every 3 min [28,33]. Combined with the dose-dependent renal reuptake, the recycling of dehydroascorbic acid to ascorbate are instrumental in maintaining vitamin C homeostasis in the body [7,44].

Parenteral administration of vitamin C bypasses the intestinal absorption and thus the saturable transport mechanism that limits the achievable plasma concentrations [[45], [46], [47]]. In contrast to oral administration, intravenous infusion of administration of 5–70 g of vitamin C produces a predictable plasma concentration and studies have shown that i. v. administration within this dose range adheres to 1st order kinetics with a constant half-life of about 2 h [48,49]. Intravenous administration of pharmacological doses of vitamin C gives rise to millimolar plasma concentrations that are not achievable by oral administration. Pharmacological doses of vitamin C are currently being evaluated in both sepsis and cancer therapy [[50], [51], [52], [53]].

## 3 Vitamin C vs. ‘normal’ low molecular weight drugs

The pharmacokinetic properties of vitamin C—as briefly outlined above—renders its dose vs concentration relationship quite different from that of a typical low molecular weight drug. Fig. 2 illustrates the differences between vitamin C and an ‘average low molecular weight drug’ with respect to plasma concentration vs time and plasma steady-state concentration vs dose as well as dependency on administration route. Elimination and steady state concentrations in tissues are illustrated in Fig. 3. Commonly, drugs display 1st order kinetics resulting in a predictable plasma and tissue concentration depending proportionally on the dose and irrespective of route of administration (Fig. 2A, B, 2E and 2F). In contrast, vitamin C shows mixed kinetics following oral administration (Fig. 2D), and mainly 1st order kinetics following intravenous administration until near-physiological levels are reached (Fig. 2C). There is a clear dose-dependency of oral administration (Fig. 2H) reaching a maximum level of about 70–80 μmol/L. Surprisingly, although displaying 1st order kinetics of over a wide range, intravenous administration may also reach a maximum level around 50 mmol/L at doses higher than 70 g/m^2^ [7]. Importantly, the data supporting the highest concentrations in Fig. 2G come from only a single study [48]. Table 1 summarizes basic pharmacokinetic properties, i.e. absorption, distribution, metabolism and excretion as well as modelling options of an average pharmaceutic drug compared to those of vitamin C. Evidently, the dose-dependency of vitamin C transport have profound impact on its pharmacology. More importantly, some essential points can be extracted from this information. Firstly, the potential efficacy of vitamin C intervention in humans is intimately linked to the vitamin C status of the individual at study start. Thus, people without some degree of vitamin C deficiency or inadequacy are very unlikely to benefit from further supplementation/intake. Secondly, multiple epidemiological studies have shown that for most parts of the World, the majority of the population ingests adequate amounts of vitamin C through their diet. Therefore, unfocussed clinical trials not using poor vitamin C status as inclusion criterion are highly unlikely to produce a measurable clinical effect. The fact that overshooting the homeostatic point of saturation around 70 μmol/L in plasma only produces a very short-lived increase in body vitamin C has been mostly ignored in the clinical literature [54]. Indeed, a re-examination of the 35 randomized controlled trials from a systematic review of vitamin C efficacy using mortality as endpoint [55] revealed that none of the studies had incorporated vitamin C status into their inclusion criteria and only one study indicated some degree of suboptimal vitamin C status prior to intervention [2].

**Fig. 3:** Comparison of vitamin C and an average low molecular weight drug with regard to tissue concentration. Plots are approximations for illustrative purposes only. **A:** Following administration, a normal drug will quickly distribute to the tissue by passive diffusion until equilibrium is reached. Subsequently, the drug is cleared from the tissue with a half-life equal to that of plasma elimination [97]. **B:** The maximal tissue concentration is proportional to the dose. **C & D:** In a vitamin C sufficient individual, tissue concentration will be at their steady state and not subject to significant fluctuation unless an insufficient dose is provided. The maximal tissue concentration of individual tissues depends on SVCT configuration and expression and display saturation kinetics with increasing doses [7,10,11]. **E:** In a vitamin C deficient individual, tissue concentrations will quickly increase when vitamin C is provided depending on SVCT2 expression and tissue priority [7]. If vitamin C administration is discontinued, the tissue concentration will gradually decline but much slower than from the plasma compartment. Some tissues such as the brain have a remarkable ability to retain vitamin C against an increasing concentration gradient as a result of emerging deficiency [92,99]. **F:** In a vitamin C deficient individual, steady state level will be reached when sufficient vitamin C is provided. Steady state concentration of the tissue does not exceed saturation level.

**Table 1:** Typical pharmacokinetic properties of an orally administered pharmaceutical drug vs. those of vitamin C obtained from food sources or supplements (modified from Refs. [3]).

Pharmacokinetic property	Typical orally administered low molecular weight drug	Vitamin C from food sources or supplements
***Absorption***	1st order absorption kinetics within the therapeutic range. Absorption through passive transport resulting in plasma concentrations in the nano- to micromolar range.	Nonlinear absorption kinetics due to a mixture of saturable active transport through SVCT1 and facilitated diffusion through GLUT transporters resulting in micromolar plasma concentrations and millimolar tissue concentrations.
***Distribution***	Primarily distributed through passive diffusion. Immediate distribution primarily determined by blood flow and tissue perfusion. Homeostasis largely based on physical-chemical properties of the drugs including lipofilicity, pKa and protein binding.	Primarily distributed through active transport. Immediate distribution based on tissue priority governed by SVCT2 transporter expression and saturation kinetics. Homeostasis depends on adequacy of dose and vitamin C status of bodily compartments.
***Metabolism***	Catabolized unspecifically by phase I & II enzymes potentially generating a range of metabolites and/or conjugates with increased water solubility.	Specifically *and* unspecifically oxidized through electron donor and antioxidant properties, respectively, but efficiently regenerated intracellularly to its reduced form by numerous cell types.
***Excretion***	Most often 1st order elimination kinetics though passive glomerular filtration and passive reabsorption depending on pKa. Overall relatively rapid excretion of parent compound and metabolites through urine and bile.	Nonlinear concentration-dependent elimination kinetics resulting in anything from 0 to 100% active renal reabsorption depending on vitamin C availability and saturation of bodily compartments.
***Modelling***	Kinetics can usually be modelled well by simple compartment and non-compartment models.	Does not comply with the basic assumption of terminal 1st order kinetics used in both compartmental and non-compartmental analysis.

## 4 Pitfalls in the design and interpretation of clinical studies of vitamin C

Several pitfalls and design challenges are involved in the assessment of the effect of vitamin C in health and disease. Some major factors have been summarized in Table 2. Epidemiological studies lack the ability to establish causal relationships and have generally not been highly valued in the hierarchy of clinical evidence. Confounding is an inheritable risk in observational studies and for micronutrient studies such as those with vitamin C, the risk of contributions from multiple or unknown deficiencies is evident and essentially impossible to definitively adjust for. Thus, identified associations between poor vitamin C status and increased risk of disease or mortality may in fact be causally related to other factors not accounted for in the study. However, in contrast to the general notion, a detailed evaluation of randomized controlled trials (RCTs) and observational studies examining the same clinical topic revealed that well-designed observational studies did not systematically overestimate the magnitude of the effects of treatment as compared with those in RCTs [56].

**Table 2:** Summary of the most important design challenges in clinical studies of vitamin C in health and disease leading to potential misinterpretation of the results and erroneous conclusions.

Study type	Design challenges	Potential pitfall in interpretation
***Observational studies***	Confounding	Vitamin C deficiency is commonly accompanied by other micronutrient deficiencies, suboptimal lifestyle and other residual confounding that may potentially contribute to or even be responsible for the observed associations.
	Using vitamin C intake as surrogate marker for vitamin C status	Vitamin C intake is a poor surrogate for vitamin C status as the estimation of vitamin C intake is inherently inaccurate and the relationship between intake and status is highly complex.
***Randomized controlled trials***	Subjects already high in vitamin C at study start	Due to the saturation kinetics of vitamin C following oral administration, individual vitamin C status greatly affect the potential effect of supplementation. As vitamin C deficiency is most commonly limited to selected subpopulations, the potential efficacy will be effectively diluted if inclusion criteria are not taking this into account.
	Placebo group continues to take supplements	Allowing continued supplement intake in the placebo group will test two doses of vitamin C against each other rather than the effect of vitamin C supplementation *per se*. Because of saturation kinetics, this will further diminish the possibility of identifying effects of the vitamin C intervention.
	Both intervention and placebo groups have had a lifelong preload with vitamin C	The human diet typically contains from 0 to 250mg vitamin C per day not considering supplementation, i.e. a wide range and with the high end being within the range or even exceeding that of several of the large intervention studies. Thus, the potential for observing disease prevention with supplementation vs placebo during the study period should be compared to the lifelong vitamin C status of all study subjects.
	Vitamin C is not tested as a single supplement	Not testing vitamin C as a single supplement limits the possibility of extracting its effect *per se*.
***All studies***	Selection bias	Recruitment may favor health-conscious, self-motivated subjects eating a healthy diet already high in micronutrients and with a lower disease rate than background population. This will limit the possibility of identifying effects of supplementation.
	Using non-fasted blood samples	Oral vitamin C intake produces a transient albeit significant increase in plasma level depending on the vitamin C status of the individual (See Fig. 2D for example). This will lead to larger variation and may result in an artefactually high average vitamin C concentration.
	Inadequate sample handling	Inadequate sampling stabilization and handling leads to increased post sampling oxidation and artefactually low vitamin C concentrations regardless of methodology.

### 4.1 Measuring vitamin C intake vs status

A possible contributor to erroneous conclusions in cohort studies is the focus on vitamin C *intake* rather than vitamin C *status*. Many cohort studies—including the largest ones—have used estimates of micronutrient intakes compiled from self-reported food frequency questionnaires (FFQs) or food diaries as their basis for correlations between vitamin C intake and disease risk (Table 3). However, as pointed out in the above, there is not a linear relationship between vitamin C intake and status. Even more importantly, the relationship between vitamin C intake and plasma/tissue homeostasis depends significantly on the vitamin C status of the individual, which is only assessable through plasma analysis. Moreover, FFQs suffer from lack of precision and accuracy due to e.g. human recall error, inability to account for vitamin loss from storage and preparation of foods as well as not accounting for polymorphisms possibly affecting vitamin C homeostasis [1,[57], [58], [59], [60]]. In order words, information from FFQs is inadequate to establish the true vitamin C status of the individual and will at the very least be encompassed with increased variability and thus increased risk of type 2 errors. Also, most cohort studies only collect information at baseline and consequently do not take changes in diet over time into account. However, plasma vitamin C status *per se* may also fluctuate considerably immediately following food or supplement ingestion [54]. Consequently, the most reliable and practically available information on vitamin C status can only be retrieved from a blood sample from a fasted individual. This requirement is clearly not met by most observational studies.

### 4.2 Instability of vitamin C

Even if fasted blood samples can be obtained, there may still be significant challenges in correlating vitamin C status to disease risk. This is due to the lability of ascorbate ex vivo. Ascorbate is quickly oxidized ex vivo and the resulting oxidation products are quickly degraded or metabolized [13], rendering the analytical recovery too low. To complicate things even more, the oxidation of vitamin C in solution is concentration dependent [61,62]. Hence, in order to obtain valid vitamin C concentrations, meticulous sample handling is critical [[63], [64], [65], [66]]. Typically, blood/plasma/serum samples retrieved from biobanks have not been specifically stabilized and stored with the intention of analyzing vitamin C and therefore not been handled appropriately to prevent post sampling oxidation. Consequently—and in this authors personal experience—generic biobank samples are rarely if ever suitable for proper quantification of vitamin C. Finally, the analysis of vitamin C has been performed by a variety of methodologies some of which are based on derivatization procedures giving rise to degradation as well as detection of a number of specimens unrelated to vitamin C. As reviewed by others, robust quantification of ascorbate is achieved by high-performance liquid chromatography using electrochemical detection [67].

### 4.3 Design problems in RCTs

RCTs are considered the gold standard for testing drug efficacy and safety. However, for testing efficacy in chronic disease prevention of micronutrients already present in the body in considerable concentrations, the RCT as design concept is subject to a number of challenges [[68], [69], [70], [71], [72]]. Micronutrient studies are most often conducted as primary disease prevention studies with lower statistical power than secondary prevention studies. Such studies may require very long intervention periods to accumulate sufficient disease endpoints [1]. This perspective may then be compared to the accumulated preventive potential of a lifelong vitamin C intake of both placebo and intervention groups up to the trial. The Nurses’ Health study collected dietary information on 85118 female nurses and estimated their diets to contain between 61 and 209 mg vitamin C/day (median intake in lowest vs. highest quintile) [73]. This suggests that a considerable proportion of the subjects recruited for intervention studies may have ingested more vitamin C than the trial supplement for many years prior to enrolment. Unfortunately, the impact of this potential bias has been completely neglected in the available literature.

Moreover, RCTs should include a placebo group. Given the challenges discussed above, it is highly questionable if this is possible in studies with micronutrients including vitamin C. In addition to this, several of the largest intervention studies with vitamin C have allowed the so-called ‘placebo group’ to continue to take supplements up to the levels of the current RDAs during the entire trial period ([[74], [75], [76]]; see Table 5). For vitamin C, this suggests that the individuals of the placebo groups could have ingested up to about 350 vitamin C mg/day and still been considered control subjects. In most cases, the frequency of concurrent supplementation in the placebo group has not been recorded but the Women's Antioxidant Cardiovascular Study reported that 27.5% of the placebo group took concurrent supplements [74]. Also from the plasma concentrations reported in the placebo group, it is apparent that the placebo group was already well within the saturation range with an average of 71.5 μmol/L [74]. As mentioned earlier, vitamin C displays dose-dependent kinetics reaching saturation around 70 μmol/L. Based on this, any significant outcome of such an intervention study would be a surprise. Effectively, intervention studies with vitamin C do not have a true placebo group but rather compare effects of two doses of vitamin C that in many cases are not very different and in terms of subject vitamin C status will result in largely overlapping populations. Collectively, this entails that the potential for intervention efficacy in these trials has generally been very low. Unfortunately, the possible benefit in individuals with poor vitamin C status at entry may therefore be diluted beyond identification.

More general challenges with clinical studies of vitamin C include the potential selection bias when people are recruited through advertisement. The “healthy enrollee effect” in micronutrient studies is well-known and describes the tendency towards recruitment of health-conscious, self-motivated subjects eating a healthy diet already rich in micronutrients and with higher exercise frequency and lower disease rate than background population [70,77]. Also, as vitamin C is highly redox active and thus a labile compound, sample handling is critical and requires special attention in particular in large multicenter trials [[63], [64], [65], [66]]. Poor attention to sample stability issues will result in lower vitamin C values due to loss during workup. In contrast, obtaining samples from individuals in the non-fasted state will result in artefactually elevated steady state levels (Table 2).

## 5 Re-examining the clinical evidence

In the following, the largest clinical studies on vitamin C are re-examined in view of the information included in Table 1, Table 2. For practical reasons, this review only reexamines the five largest studies in each category. These studies may be considered the most influential in terms of authoritative impact and serves to illustrate the challenges in the literature on vitamin C rather than providing an exhaustive systematic review.

### 5.1 Prospective cohort studies estimating vitamin C intake

A considerable number of observational studies have examined the relationship between vitamin C and morbidity and mortality for decades. The largest of all studies of vitamin C and disease are all cohort studies estimating disease risk/mortality in relation to vitamin C intake using FFQs and food diaries rather than by measuring vitamin C status *per se*. Consequently, they all suffer from the problems in relating estimated intake to actual vitamin C status of the individual. The studies are listed in Table 3.

**Table 3:** Effect of vitamin C intake on disease risk/mortality in major observational studies. Major limitations of the presented studies are that i) they estimate vitamin C intake as surrogate for vitamin C status, ii) most studies suffer from selection bias and iii) only a single estimate of vitamin C intake is used.

Survey Data	The Nurses' Health Study [73]	Etude Epidémiologique aupre's de femmes de la Mutuelle Générale de l’Education Nationale [78]	*The Health Professionals* Follow-up Study [79]	EPICOR Study [80]	Iowa Women's Health Study [81]
***Study Population***	85,118 healthy US female nurses, aged 30–45 yrs	57,403 French healthy women, aged 40–65 yrs	43,738 US men w/o CVD or diabetes, aged 40–75 yrs	41,620 Italian men & women w/o MI or stroke, aged 44–61 yrs	34,492 US postmenopausal women, aged 55–69 yrs
***Highest median vitC intake (mg/d)***	704; top quintile	228^a^; top quartile	1167; top quintile	201; top tertile	679; top quintile
***Lowest median vitC intake (mg/d)***	70; bottom quintile	77.5^a^; bottom quartile	95; bottom quintile	83; bottom tertile	82; bottom quintile
***Adjustments***	Age, energy intake, supplements use, alcohol, smoking status, and diabetes	Age, oral contraceptives, hormone therapy, alcohol, BMI, physical activity, energy intake, smoking, supplement use, education, and specific breast cancer risk factors	Age, season, smoking, energy intake, alcohol, hypertension, parental history of MI, profession, BMI and physical activity.	Age, center, sex, hypertension, smoking, education, energy intake, alcohol, waist circumference, obesity, and physical activity.	Age, BMI, waist-to-hip ratio, hypertension, diabetes, ERT, education, marital status, smoking, physical activity, energy intake, cholesterol, alcohol, saturated fat, fish, vitE, carotenoids, fiber, and whole grains
***Follow-up period (years)***	16	10	8	7.9	11
***Endpoint***	CHD	Postmenopausal breast cancer	Stroke	Stroke	Death from stroke
***Outcome***	Inverse association between vitC intake and risk of CHD. VitC supplementation was associated with lower risk of CHD	VitC supplement use not associated with breast cancer risk; Top quartile of vitC intake from foods only showed increased risk of breast cancer	Neither vitC intake nor supplementation was associated with lower risk of stroke	VitC associated with lower risk of ischemic stroke	No association between vitC intake and death from stroke

Abbreviations: BMI, body mass index; CHD, chronic heart disease; CVD, cardiovascular disease; DBP, diastolic blood pressure; ERT, estrogen replacement therapy; IHD Ischemic heart disease; MI, myocardial infaction; SBP, systolic blood pressure; vitC, vitamin C; vitE, Vitamin E. ^a^Reported as mean intake from food only.

The Nurse’ Health Study examined the association between vitamin C intake and supplementation on the risk of chronic heart disease [73]. They found both a significant inverse correlation between vitamin C intake and chronic heart disease but also a positive association to supplement use. A semi-quantitative FFQ was used to assess micronutrient intake including supplements four times during the follow-up period. As acknowledged by the authors, a major weakness of the study was that the population was well-nourished as shown e.g. by the estimated median vitamin C intake of the non-supplement users of 132 mg/day, which amounts to more than twice the RDA at the time of the study. Thus, the study does not provide insight to the possible benefit in individuals with low vitamin C status or risk factors of CVD.

The French E3N study assessed the possible association between estimated vitamin C intake from both food and supplements and risk of postmenopausal breast cancer in a cohort of healthy women primarily comprising teachers [78]. The study found no overall association between vitamin C supplementation and breast cancer but surprisingly, the top quartile of vitamin C intake from food only showed increased risk of breast cancer suggesting a possible U- or J-shaped relationship. A self-developed FFQ was used to estimate nutrient intake and in a validation study not described in detail, the correlation coefficients for vitamin C intake were 0.73 for reproducibility and 0.55 for validity, which is rather low. Unfortunately, the FFQ was not validated towards vitamin C status as thus not particularly well suited for this purpose. Whereas vitamin C supplementation was assessed several times through follow-up, the estimated vitamin C intake from food was only estimated at a single baseline time-point. Thus, a part from the limitation of being based on FFQs, the study does not account for any dietary changes over the 10 year follow-up period.

In the Health Professionals Follow-up Study [79], the possible relationship between estimated vitamin C intake and risk of stroke was examined in healthy men. The study reported no association between either vitamin C intake or supplementation and risk of stroke after eight years. Vitamin C intake from food and supplements was assessed biannually using FFQs. As with the studies mentioned above—and as acknowledged by the authors—this population was better nourished than the average population and thus, the study does not provide much insight to the possible benefit in individuals with poor vitamin C status or risk factors of stroke and CVD.

The EPICOR study represents the Italian segment of the European Prospective Investigation into Cancer and Nutrition (EPIC) study cohort and investigated the possible correlation between estimated vitamin C intake and ischemic stroke [80]. The study found that vitamin C was significantly associated with decreased risk of ischemic stroke. The study used an estimated total antioxidant capacity as the primary outcome and thus, correlations with vitamin C intake was the results of a sub-analysis. Total antioxidant capacity is a very crude measure—and in this case an indirect estimate—of countless more or less important molecules displaying antioxidant activity. While it may possible be considered a surrogate marker of fruit intake, many other components including coffee and wine were also showed to contribute considerably [80]. A severe weakness of the study is the very low number of total stroke cases amounting to only 194 per 328,553 person years examined. Moreover, the estimated vitamin C intake was only estimated once at baseline. Consequently, the study does not account for any dietary changes over the almost 8 year follow-up period.

The Iowa Women's Health Study assessed the possible correlation between estimated vitamin C intake and mortality from stroke in postmenopausal women [81]. No association between vitamin C intake and death from stroke was observed. The study population was part of a random sample of Iowa women with driver's license. The validity of the FFQ also used in the in the Nurses' Health study mentioned above [73] was done by comparing mean intakes from five 24-h dietary recalls with responses from the food-frequency questionnaire in a subgroup of 44 women [82]. Consequently, they were not assessed for correlation to plasma vitamin C status. The correlation coefficients for the comparison of the two methods of diet assessment for intakes of vitamin C was 0.53 for food only and 0.76 for combined intake from food and supplements [81]. Again, only one estimate at baseline was performed.

Collectively, the above studies are all very large and with considerable follow-up periods. However, they were all designed as broad purposed population surveys without the specific intention of studying effects of vitamin C intake. The three largest studies have clear selection bias towards well-nourished individuals, i.e. health care professionals and teachers. This severely limit their usefulness in identifying associations between vitamin C status and disease, as vitamin C intake above average has very little impact on systemic vitamin C status. Also most of them only included a single baseline estimate of vitamin C intake, which may seriously misrepresent dietary patterns and changes during the study period but even more importantly also the life-long dietary habits leading up to the study that could potentially have a stronger impact on disease risk. Finally, the potential for residual confounding with regard to vitamin C is expectedly relative high, as the correlation between vitamin C intakes and status is low particularly at high intakes.

### 5.2 Observational studies measuring vitamin C status

Limiting the examination to studies measuring blood vitamin C status rather than estimating vitamin C intake using FFQs or food diaries should, at least in theory, improve the scientific quality considerably. These studies are summarized in Table 4. The EPIC-Norfolk survey have given rise to a considerable number of studies including two on vitamin C [83,84]. Both prospective cohort studies included about 20,000 men and women. The first study examined the possible relationship between all-cause, cardiovascular disease, ischemic heart disease and cancer mortality after four years [84]. The study showed that vitamin C status was significantly inversely correlated to all-cause mortality as well as mortality due to cardiovascular disease and ischemic heart disease. The data also revealed a clear concentration-response relationship: For each 20 μmol/L rise in plasma vitamin C concentration, a 20% reduction in risk of all-cause mortality could be observed (p<0·0001). The risk of death was about half in the top compared to bottom quintile with respect to vitamin C status. The findings are impressive considering the short follow-up period of only four years. However, as with most of the previously mentioned studies, vitamin C (status in this case) was only assessed a single time at baseline. With the short duration though, chances of markedly changed dietary habits diminishes but are still relevant. Moreover, the study did not adjust for social class and physical activity as these data were not available at the time of analysis. The second EPIC-Norfolk investigated the relationship between plasma vitamin C status and risk of stroke with a follow-up period of nearly ten years [83]. The study found a 42% lower risk of stroke in the top compared to bottom quartile of vitamin C status. The study was based on 448 incidents of stroke per 196,713 person years, i.e. about a 4-fold higher incidence than in the EPICOR study mentioned above. Both studies quantified vitamin C using a fluorometric assay after derivatization. These assays are known to have less accuracy and precision than methods based on high-performance liquid chromatography [67]. However, if meticulous sample handling has been applied, a general over or underestimation of samples would not affect the study outcome and the potentially increased variation would only attenuate the significance of the differences observed. Both studies used non-fasted blood samples, which generally overestimates vitamin C status.

**Table 4:** Effect of vitamin C status on disease risk/mortality in major observational studies. Limitations of the presented studies are that they i) used non-fasted blood samples, ii) less than optimal analytical methodology and iii) do not account for possible multi-deficiencies.

Survey Data	EPIC-Norfolk [83]	EPIC-Norfolk [84]	NHANES II [85]	NHANES II [87]	NHANES II [86]
***Study Population***	20,649 men and women from Norfolk, UK, aged 40–79 yrs	19,496 men and women from Norfolk, UK, aged 45–79 yrs	8417 US men and women, aged 30–75 yrs	7071 US men and women aged 30–75 yrs	6624 US men and women aged 40–74 yrs
***Highest group vitC conc (μmol/L)***	≥66.0; top quartile	79.2; top quintile	79.5 (64.7–158.8)	≥73.8; top quartile	85.2 (64.7–158.8)
***Lowest group vitC conc (μmol/L)***	<41.0; bottom quartile	25.9; bottom quintile	17.0 (5.7–22.7)	<28.4; bottom quartile	17.0 (5.7–22.7)
***Fasted blood samples (Yes/No)***	No	No	No	No	No
***Method of analysis***	Fluorometric assay	Fluorometric assay	Colorimetric assay	Colorimetric assay	Colorimetric assay
***Adjustments***	Age, sex, smoking, BMI, SBP, cholesterol, physical activity, diabetes, MI, social class, alcohol & supplement use	Age, systolic blood pressure, cholesterol, smoking, diabetes, & supplement use	Gender	Smoking status	Age, sex, race, education, physical activity, smoking, alcohol, cholesterol, BMI, diabetes, hypertension, aspirin and vitE use
***Follow-up period (years)***	9.5	4	?*	12–16	?*
***Endpoint***	Stroke	All-cause, CVD, IHD and cancer mortality	All-cause, CVD and cancer mortality	Cancer & all-cause mortality	CVD
***Outcome***	Risk of stroke was 42% lower in top vs bottom quartile	VitC inversely related to all-cause, CVD & IHD death. Risk of death was about half in top vs bottom quintile	Mid and top vitC groups had 25–29% decreased risk of all-cause mortality compared to bottom vitC group	Men in bottom vs top quartile had 57% increased risk of all-cause mortality & 62% higher risk of cancer death	Serum vitC independently associated with CHD & stroke; 27% lower risk in top vs bottom group

Abbreviations: BMI, body mass index; CHD, chronic heart disease; CVD, cardiovascular disease; IHD, Ischemic heart disease; MI, myocardial infaction; SBP, systolic blood pressure; vitC, vitamin C; vitE, Vitamin E. *Follow-up period not specifically specified.

Data from the Second National Health and Nutrition Examination Survey (NHANES II) were used as basis for the following three studies. Simon et al. examined the relationship between serum ascorbic acid and cause-specific mortality [85]. They reported a trend towards decreased risk of CVD in people with normal or high compared to low vitamin C levels and a 25% decreased risk of all-cause mortality. From another NHANES II study, they concluded that serum vitamin C status was independently associated with lower risk of stroke and chronic heart disease [86]. A non-linear concentration-response relationship between vitamin C concentration and risk of both conditions was found with an expected particular higher effect of vitamin C deficiency. Loria et al. examined the same cohort and found that the bottom quartile of serum vitamin C levels had 57% increased risk of all-cause death and 62% increased risk of cancer death compared to the top quartile [87]. While Simon et al. reported a significantly lower cancer risk in men with high vitamin C status, they unexpectedly found a higher risk in women with high levels of vitamin C [85]. However, this difference was not observed by Loria and coworkers using the same cohort [87]. All the studies assessed vitamin C in serum from non-fasted blood samples using a colorimetric assay.

Collectively, the above studies are large with mixed follow-up periods. They appear to have less selection bias than the FFQ based studies discussed above. Interestingly, all studies found a significant relationship between high vitamin C status and decreased risk of morbidity or mortality. Thus, a potential selection bias towards healthy enrollees would likely have attenuated the effect. However, the five studies are based on only two different population surveys and therefore essentially only represent two separate studies. All studies suffer from less than optimal analytical methodology, in part explainable by the very large number of samples and era of analysis, but potentially leading to increased risk of over- or under-estimation of vitamin C. They have all used non-fasted blood samples as basis for the vitamin C measurement generally leading to an overestimation of the vitamin C status. Also, they do not account for possible confounding from potential multiple micronutrient deficiencies that could impact the relevance of the correlations.

### 5.3 Randomized controlled trials using vitamin C in the intervention

#### 5.3.1 The Linxian study

The major RCTs using vitamin C in their intervention are summarized in Table 5. The Linxian study was the first major RCT to study the effect of antioxidant and mineral intervention [88]. The setting of Linxian, China, was chosen because of its high esophageal cancer rate and poor general nutritional status of the population. In a complex ½ (2 × 2 x 2 × 2) design, the authors aimed to test the combined effect of nine vitamins and minerals in a fractional design, where all participants received one of seven combinations of four grouped supplements or placebo for 5.25 yrs. The vitamin C supplement (120 mg/day) was combined with Molybdenum (30μg/day). No effect of vitamin C and molybdenum was observed on mortality and cancer incidence [88]. Baseline vitamin C levels were assessed 10 months prior to study start in 49 individuals allocated to supplements and 49 allocated to placebo both of which indicated severe vitamin C deficiency, however, with intervention group participants being significantly lower than placebo (p<0.03). A blood sample during the intervention trial was obtained from 730 to 740 individuals from intervention and placebo groups, respectively. Expectedly, the vitamin C status improved significantly over placebo to 46 μmol/L in the intervention group (p<0.001) but surprisingly, the vitamin C status of the placebo group also showed a highly significant increase to 30.7 μmol/L from baseline (p<0.001), indicating that both groups were in the suboptimal range at this point [2] and clearly increased from study start. It was not reported if the placebo group was allowed to take concurrent supplements but considering their suboptimal status, supplement use is probably unlikely to have been widespread. The Linxian study is interesting as it is the only major RCT that have allegedly included vitamin C deficient subjects. However, the significantly increased vitamin C status in the placebo group raises serious concerns. This suggests either that the baseline levels were severely underestimated in the very small sample of individuals analyzed at study start, *e.g.* by coincidence, poor analytical methodology or inappropriate sample handling, or that the placebo group improved their diet during intervention, *e.g.* by diet change or concurrent supplementation. Regardless of the reason, the change in the placebo group severely limits the study's ability to assess the effect of the vitamin C intervention. Another major concern is the amount of vitamin C in the supplement. At the time of the study, the RDA for vitamin C was 60 mg/day and the supplement included twice that amount, i.e. 120 mg/day. It appears highly questionable if such a limited amount of vitamin C—which was clearly insufficient to normalize the vitamin C status of the intervention group—could be expected to result in a change in morbidity or mortality over a time span of only 5 years compared to the impact of a presumed life-time of severe vitamin C deficiency. Also, a 25-year post-trial follow-up of the trial expectedly showed no effect of the 5.25 year supplementation period [89].

**Table 5:** Effect of vitamin C supplementation in major randomized controlled trials. Major limitations of the presented studies are that they mostly i) allowed concurrent supplementation in the placebo group, ii) included vitamin C sufficient individuals and iii) used multi-vitamin supplements with inadequate amounts of vitamin C.

Study	Linxian Study [88]	Heart Protection Study [75]	Physicians Health Study II [76]	SU.VI.MAX Study [90]	Women's Antioxidant Cardiovascular Study [74]
***Population***	29,584 men and women from Linxian County, Henan Province, China, aged ≥40 yrs	20,536 British men and women aged ≥40 yrs with CHD or other occlusive arterial disease or diabetes	14,641 US male physicians age ≥50 yrs	13,017 French men and women aged ≥35 yrs	8171 US women aged ≥40 yrs and with prior CVD or high risk
***Design***	½ (2 × 2 x 2 × 2)	2 × 2	2 × 2 ( × 2 × 2)	Parallel	2 × 2 × 2
***VitC conc at entry (μmol/L)***	11.4^a^	Not reported	Not reported	54.5	Not reported
***VitC conc in placebos (μmol/L)***	30.7	43.2	Not reported	58.0	71.5
***VitC group vs placebo (Δμmol/L)***	15.3	+15.7^b^	Not reported	+11.3^c^	+35.2^d^
***Fasted blood samples (Yes/No)***	Not reported	No	Not reported	Yes	Not reported
***Subjects allowed to take concurrent supplements (placebos taking suppl.)***	Not reported	Yes, but not high dose vitE (Not reported)	Yes, up to the RDA (4.4% for 1 month/yr or more)	No	Yes, up to the RDA (27.5%)
***Intervention***	Various vitamin/mineral combinations including Vitamin C (120 mg/d) + Mo	Multivitamin containing Vitamin C (250 mg/d)	Vitamin C (500 mg/d) or other antioxidants	Multivitamin containing Vitamin C (120 mg/d).	Vitamin C (500 mg/d) or other antioxidants
***Study period (years)***	5.25	5	8	7.5	9.4
***Endpoint***	Mortality and cancer incidence	Major coronary events and fatal or non-fatal vascular events	Cardiovascular events, myocardial infarction, stroke, or CVD death	Ischemic cardiovascular disease and all-cause mortality	Myocardial infarction, stroke, coronary revascularization, or CVD death
***Outcome***	No effect of vitamin C + Mo supplementation	No effect of vitamin C supplementation	No effect of vitamin C supplementation	No effect on CVD but lower all-cause mortality in men	No effect of vitamin C supplementation

Assessed in ^a^98 individuals, ^b^about 5% of the participants, ^c^an unselected subsample, ^d^30 local participants. Abbreviations: CVD, cardiovascular disease; Mo, molybdenum.

#### 5.3.2 The British Heart Protection Study

The British Heart Protection Study investigated the effect of a multivitamin supplement containing 600 mg vitamin E, 250 mg vitamin C, and 20 mg β-carotene daily vs placebo for five years in a high risk population of men and women with coronary disease, other occlusive arterial disease, or diabetes in a 2 × 2 design also including simvastatin [75]. No significant reductions in the 5-year mortality from, or incidence of, any type of vascular disease, cancer, or other major outcome were observed from the antioxidant intervention. Vitamin C status was not measured at study start but judging from the assessment of vitamin C status in non-fasted blood samples at follow-up—carried out in about 5% of the participants—the participants were not vitamin C deficient prior to supplementation. However, the intervention did produce a significant 15.7 μmol/L increase in vitamin C status compared to placebo, 58.9 vs 43.2 μmol/L. The methodology used for vitamin C determination or sample handling is not reported. All participants were allowed to continue any prior supplement use during the study period except for high dose vitamin E. The number of concurrent supplement users in each allocation group was not reported. From the use of non-fasted blood samples, the vitamin C status of the study population is likely somewhat overestimated. In spite of this, it is worth noticing that the vitamin C supplement used was clearly insufficient to saturate those allocated to intervention, thus resulting in partly overlapping populations. Again, the relatively short duration and modest size of the intervention has to be compared to the high-risk status of the study population and their life-time dietary and supplement history that is not known or accounted for in order to judge if it is reasonable to expect a study effect under these conditions. Based on the available information, this appears highly questionable.

#### 5.3.3 The Physician's Health Study II

The Physician's Health Study II RCT investigated the effect of eight years of supplementation with vitamin C (500mg/day) and vitamin E (400IU every other day) vs placebo on cardiovascular disease risk in 14641 male physicians aged ≥50 years in a 2 × 2 design [76]. Vitamin C supplementation did not reduce the risk of major cardiovascular events in this period. The vitamin C status of the study participants was not assessed either at entry or during or post intervention. This seriously limits the possibility of reexamining and concluding on the data, as the potential effect of the 500 mg/day vitamin C supplementation on the vitamin C status of the individual may vary from highly significant to negligible depending on their entry level and dietary habits. Also, a potential bias between groups cannot be excluded. Furthermore, the study participants were allowed to take concurrent supplements up to the RDA during the trial. Concurrent supplement use was reported only if used for more than a month per year. These numbers were only 4.4% among the placebos.

#### 5.3.4 The SU.VI.MAX study

The SU.VI.MAX study was carried out in French men and women slightly younger than those of the other studies (≥35 yrs) [90]. The study tested the efficacy a daily multivitamin and mineral supplement containing nutritional doses of vitamin C (120 mg), vitamin E (30 mg), β-carotene (6 mg), selenium (100 μg) and zinc (20 mg) vs placebo in a parallel design for 7.5 years in reducing the incidence of cancer and ischemic heart disease in the general population. Although the study showed no significant effect on the main outcome, a sub analysis did reveal a significant positive effect of supplementation on cancer incidence [p<0.008) and all-cause mortality (p<0.02) in men [90]. The authors attributed this gender effect to the generally lower vitamin C status among men. Vitamin C status at entry was assessed in fasted blood samples from ‘an unselected subsample’ and showed that participants were adequate although not entirely saturated with vitamin C at entry. Intervention produced a slight albeit significant increase in plasma vitamin C status compared to placebo and the placebo group was not allowed to take concurrent supplements. Although carefully designed with respect to several of the pitfalls mentioned earlier, the present study has several shortcomings in terms of investigating the potential of vitamin C supplementation on human disease risk. Thus, the serious selection bias in terms of well-nourished individuals with a relatively high vitamin C status combined with the low-dose supplement limits the likelihood of identifying an effect of supplementation. The 120 mg vitamin C per day provided in the supplement has probably been close to or less than that ingested through the diet of the study participants in general. Moreover, the positive effect observed in men cannot be directly attributed to the vitamin C supplementation as vitamin C was not provided as a single supplement. In spite of these limitations, the SU.VI.MAX study adequately demonstrates that limited if any effect of low-dose supplementation can be expected in already well-nourished individuals with an adequate vitamin C intake. However, it would have been highly interesting had the study been conducted in a vitamin C deficient population with a 500–1000 mg/day vitamin C supplement.

#### 5.3.5 The Women's Antioxidant Cardiovascular Study

The final major intervention study using vitamin C reexamined here—The Women's Antioxidant Cardiovascular Study—investigated the effects of ascorbic acid (500 mg/d), vitamin E (600 IU every other day), and beta carotene (50 mg every other day) on the combined outcome of myocardial infarction, stroke, coronary revascularization, or CVD death among 8171 female health professionals 40 years or older at increased risk of CVD in a 2 × 2 x 2 factorial design for 9.4 years [74]. The study found no overall effects of vitamin C, vitamin E, or beta carotene on cardiovascular events. Vitamin C status of the study population was not recorded at entry. Judging from the assessment in ‘30 local participants' about halfway through the study [74], the study population—including the placebo group—was saturated in vitamin C throughout the study. Although not reported in the paper, it would appear from the high vitamin C status (in particular in the intervention group) that fasted blood samples were clearly not obtained. Also, concurrent supplement use up to the RDA was allowed in the study population and 27.5% of the placebo group reported taking supplements during the trial. In spite of the amount of vitamin C provided as supplement in the present study, the inadequate inclusion and exclusion criteria used only allows for the conclusion that additional vitamin C supplementation to already saturated high-risk individuals does not provide further protection from CVD.

Collectively, the above studies suffer from serious deficiencies preventing them from drawing relevant conclusions on the potential benefit of vitamin C supplementation in particular in populations with poor vitamin C status. All except one study allowed the placebo group to take concurrent supplements and three of the five examined only the combined effect of a multivitamin cocktail with low dose vitamin C. Study placebo participants mostly showed adequate to saturated levels of vitamin C if measured and in the Linxian study that supposedly examined a population with poor nutrition, vitamin C levels almost tripled in the placebo group during the study (Table 5).

## 6 Concluding remarks

As exemplified above, clinical studies examining the relationship between vitamin C and health, disease and mortality—or indeed the effect of supplementation—generally suffer from many limitations that seriously impair their ability to draw conclusions on the importance of vitamin C in human health. In epidemiological studies, a baseline assessment of vitamin C status may represent the lifestyle of the individual and thus be an indication of life-long exposure, although this is far from certain as diet changes are not accounted for. In intervention studies, the intervention arm(s) represent a *change* in lifestyle, the impact of which has to be compared to that of the life-long exposure prior to the intervention. In that perspective, the intervention periods and doses appear completely inadequate to robustly identify a putative benefit of supplementation, in particular when looking at populations that are not low or deficient in vitamin C. Thus, when reexamining the clinical literature on vitamin C, one is left with little certainty and many questions, including those presented in the introduction: *What is the optimal intake of vitamin C and what is its preventive and therapeutic potential?*

Collectively, there seems to be a relatively persistent association between poor vitamin C status and increased risk of disease and premature death. However, it is not known if this increased risk of morbidity and mortality from vitamin C deficiency is a result of lack of vitamin C *per se*, multiple co-deficiencies or deficiencies in other substances than vitamin C. The intervention studies may serve to demonstrate that supplementation with vitamin C to already saturated individuals apparently has little or no effect on morbidity and mortality. However, it remains unknown if supplementation with vitamin C to individuals with poor vitamin C status can prevent disease development or progression. A possible way of adding new information to this complex issue could be to recruit individuals with genetically unfavorable SNPs in SVCTs. These individuals are likely to represent a life-long poorer vitamin C status without abundant co-deficiencies. Consequently, it would be possible study their risk of vitamin C deficiency attributable diseases. However, as it is probably not possible to counteract the negative effect of a SNP lowering the vitamin C homeostasis by supplementation, these individuals are not particularly suited for intervention studies. A major challenge with this type of studies is that the frequency of these SNPs is very low resulting in relatively low power in spite of enormous populations. Thus, well-designed studies are (still) needed to explore the putative role of vitamin C deficiency in disease development and progression and the potential benefit of supplementation to individuals with poor nutritional status.

Finally, biological signatures for vitamin C action, i.e. biomarkers or combination of biomarkers that specifically and robustly reflect a condition, are desperately needed to improve the assessment of physiologically sufficient/insufficient vitamin C status and the potential concentration-response relationship between vitamin C status and specific diseases. So far, very limited knowledge is available on the relationship between vitamin C status and the function of the individual physiological processes for which vitamin C provides the reducing equivalents in vivo. From animal studies, it is known that a ‘hierarchy’ of the tissues/organs exists that determines which part of the body that get the vitamin C if limited resources are available [26,27,31,[91], [92], [93]]. These show that e.g. the brain is clearly prioritized during periods with inadequate supply of vitamin C. Importantly, such prioritization may have serious implications for the clinical effect of vitamin C deficiency and suboptimal vitamin C status. Thus, very limited amounts of vitamin C are necessary to prevent scurvy, suggesting a highly favorable concentration/response relationship for the underlying physiological mechanisms. However, the potential prioritization between the vitamin C dependent processes required to maintain e.g. cardiovascular function, immune system and neuronal health remains unknown. The elucidation of such disease specific concentration-effect relationships require highly robust biological signatures not yet available.

## Declaration of competing interest

None.
